# Experimental Study on the Correlation between miRNA-373 and HIF-1*α*, MMP-9, and VEGF in the Development of HIE

This article has been retracted.

**DOI:** 10.1155/2021/5553486

**Published:** 2021-05-03

**Authors:** Chun-Yang Liu, Hisham Al-Ward, Francine Ngaffo Mekontso, Ning Liu, Hui-Qin Zeng, Min Liu, Zi-Rui Yu, Lin Zhang, Yu-Chun Han, Hui Xu

**Affiliations:** ^1^Department of Biochemistry and Molecular Biology, Jiamusi University School of Basic Medical Sciences, Jiamusi, China; ^2^AnKang University, School of Medicine, Ankang, Shanxi Province 725000, China; ^3^Hainan University, Haikou, Hainan Province, China; ^4^First Affiliated Hospital of Xiamen University, Xiamen 361003, China; ^5^Beijing Friendship Hospital, Capital Medical University, Beijing 100000, China; ^6^Inner Mongolia Medical University, Hohhot, Inner Mongolia, China; ^7^Jiamusi University, School of Clinical Medicine, Jiamusi, China

## Abstract

**Introduction:**

Microribonucleic acids (miRNAs) have short (approximately 18 to 25) nucleotides and are evolutionarily conserved and endogenously expressed RNAs belonging to a family of noncoding RNA molecules. miRNA-373 regulates cell proliferation, migration, apoptosis, invasion, and repairing damaged DNA after hypoxia stress. Neonatal hypoxic–ischemic encephalopathy (HIE) refers to perinatal asphyxia caused by partial or complete hypoxia, reduced or suspended cerebral blood flow, and fetal or neonatal brain damage. We aim to investigate the relationship between miRNA-373 and HIF-1*α*, between miRNA-373 MMP-9, and between miRNA-373 VEGF in the occurrence and development of HIE.

**Methods:**

Human (children) samples were divided into four groups (*n* = 15 in each group) according to HIE severity. The patient group was divided into middle, moderate, and severe HIE groups. The control group included healthy children or children with nonneurological diseases. The expressions of miRNA-373, HIF-1*α*, MMP-9, and VEGF were assayed in the serum samples.

**Results:**

Our study showed a strong relationship between miRNA-373 and HIF-1*α*, between miRNA-373 and MMP-9, and between miRNA-373 and VEGF. The expression levels of miRNA-373, HIF-1*α*, MMP-9, and VEGF in the HIE groups were much higher than those of the control group.

**Conclusion:**

The increased change in miRNA-373 expression has a certain diagnostic significance on neonatal HIE. In the occurrence and development of HIE, miRNA-373 is positively correlated with HIF-1*α*, MMP-9, and VEGF.

## 1. Introduction

Neonatal hypoxic–ischemic encephalopathy (HIE) refers to perinatal asphyxia caused by partial or complete hypoxia, reduced or suspended cerebral blood flow, and fetal or neonatal brain damage. As HIE is the cause of neonatal brain damage, it is also one of the important causes of death. According to statistics, the annual rate of asphyxia among newborns in China is from 6% to 15%, and between 20% and 40% die from asphyxia during the neonatal period. Approximately 200,000 children have varying degrees of disability, and some of them have permanent neuropsychiatric disorders. The degree and location of severe sequelae in hypoxia, including cerebral palsy, limb paralysis, visual and auditory impairment, motor cognitive impairment, and mental retardation, are seldom investigated, hence the massive impact on families and the society [1]. HIE currently accounts for 23% of all neonatal deaths worldwide [2]. Thus far, the medical communities in China and overseas have no unified understanding of the HIE's causes, and no effective treatment method is currently available [1]. Therefore, in-depth investigations and analyses of the risk factors and molecular biological mechanisms of neonatal HIE are necessary. Furthermore, highly effective clinical treatment methods should be sought in the field of HIE.

Micro ribonucleic acids (miRNAs) have short (approximately 18–25) nucleotides and are evolutionarily conserved and endogenously expressed RNAs belonging to a family of noncoding RNA molecules. Thousands of new miRNAs are found in different organisms every year [3]. Thus far, more than 38,589 miRNAs with diverse functions have been discovered. miRNA regulates gene expression at the posttranscriptional level. Many pathological conditions are caused by the imbalance of miRNAs [4–6], including neurodegenerative diseases, inflammatory diseases, metabolic diseases [7], cardiovascular diseases, and cancer [8, 9]. Changes in microRNA expression are closely related to the occurrence, invasion, metastasis, and drug resistance of cancer cells [10, 11].

Studies have shown that miRNA-373 is related to HIF-1*α*, MMP-9, and VEGF, as well as all hypoxic diseases, but the correlations between the aforementioned four molecules remain unclear. In this study, the correlation between miRNA-373 and HIF-1*α*, between miRNA-373 MMP-9, and between miRNA-373 VEGF are experimentally investigated and comprehensively analyzed by using bioinformatics.

## 2. Methods

### 2.1. Collection of Samples

The study subjects were children with HIE treated in the Department of Neonatology at the First Affiliated Hospital of Jiamusi University between January and June 2019. The samples were divided into four groups (15 samples in each group) according to the disease's severity, namely, the middle HIE, moderate HIE, severe HIE, and control groups. The samples in the control group were healthy children or children with nonneurological diseases who have undergone physical examination at the same time. All procedures performed in this study accord with the ethical standards of the Institutional Research Committee and the 1964 Helsinki Declaration and its subsequent amendments or comparable ethical standards. Informed consents were obtained from the parents of all participants. The study was approved by the Human Research Ethics Committee of Jiamusi University (No. JD10002).

### 2.2. Real-Time Quantitative PCR

Total RNA was extracted from serum samples by using the miRamp kit (TianGenBiotech Co., Beijing, China). Then, cDNA was synthesized using the miRcute Plus miRNA First-Standard cDNA kit (TianGenBiotech Co., Beijing, China). SYBR Green miRcute Plus miRNA qPCR Kit (TianGenBiotech Co., Beijing, China) was used to perform real-time PCR. The levels of PCR products were normalized with housekeeping U6. The relative quantitative level of miRNA-373 was determined by means of the RQ = 2^−ΔΔCt^ method.

### 2.3. ELISA

The protein levels of HIF-1*α*, MMP-9, and VEGF in the samples were measured using human ELISA kits according to the manufacturer's instructions (Shanghai Enzyme-Linked Biotechnology Co., Shanghai, China).

### 2.4. Statistical Analysis

Data analysis and graph plotting were conducted using the SPSS 19.0 (SPSS Inc., Chicago, IL, USA) software. The results were expressed as mean ± SDEV. Then, *t*-test followed by one-way ANOVA were used for data analysis. The statistical significance was defined as *P* < 0.05.

## 3. Results

The total RNA of a research subject's serum sample was extracted, and a nucleic acid quantifier was used to determine RNA concentration and purity. The optical density (A260/A280) was between 1.8 and 2.0. The RNA was not degraded, and the quality was good.

After the reverse transcription of RNA to generate cDNA, agarose gel electrophoresis was performed. The electrophoresis results are shown in Figure 1. Then, fluorescence quantitative PCR detection was conducted. The melting curve analysis did not show any spurious peaks, indicating that the amplified product was single without nonspecific amplification. The amplification curve also showed that all samples have entered the amplification plateau phase, indicating that the reaction conditions had been set accurately (Figure 2).

U6 was used as the internal control. The Ct value (i.e., the number of cycles experienced when the fluorescence signal in each reaction tube reaches the set threshold) was automatically calculated after the reaction. Each reaction tube's Ct value was logarithmically and linearly related to the initial copy number of the template. The smaller was the Ct value, the higher is the initial copy number of the gene, and the higher is the gene expression. For the comparison of 2^-*ΔΔ*Ct^ values of each group in the fluorescence quantitative PCR detection, the 95% confidence interval method was adopted. The Ct values of miRNA-373 and U6 according to the amplification curve were determined by means of the *Δ*Ct (ΔCt = CtmiRNA^∗^ − CtU6) method. The 2^-*ΔΔ*Ct^ method was used to compare the expression levels of miRNA-373 between the case group and the control group. The findings showed that the expression level of miRNA-373 in the case group was higher than that in the control group (*P* < 0.05) Figure 3.

The ELISA method was used to detect the HIF-1*α*, MMP-9, and VEGF. The values of HIF-1*α*, MMP-9, and VEGF in each subgroup of the case group were significantly increased, and the differences were statistically significant compared with those of the control group (*P* < 0.01) (Figures 4–6).

Then, a correlation analysis of patient (human) sera was performed on the basis of the miRNA-373 and HIF-1*α*, MMP-9, and VEGF. Hierarchical clustering and heatmap analysis were also conducted. Finally, Pearson correlation coefficient methods were performed to analyze the results. The findings indicate that the patient (human) sera, i.e., between miRNA-373 and HIF-1*α*, between miRNA-373 and MMP-9, and between miRNA-373 and VEGF, were positively correlated with coefficients of 0.94, 0.92, and 0.945, respectively. The closer is the correlation coefficient to 1, the stronger is the positive correlation. The results of the correlation analysis further indicate that the aforementioned four molecules have strong positive correlations. Therefore, when the miRNA-373 expression increases, the expressions of HIF-1*α*, MMP-9, and VEGF also increase, and the difference is statistically significant (*P* < 0.05), as shown in Figure 7.

## 4. Discussion

As the pathogenesis of HIE is still unclear, the correlation between the related molecules detected in the HIE should be studied to be able to further determine its pathogenesis. Relevant studies have confirmed that miR-373 regulates cell proliferation, apoptosis, senescence, mesendoderm differentiation, migration and invasion, and other processes. HIE also participates in hypoxia response and participates in DNA damage repair in the form of hypoxia-induced miRNA. miRNA-373 is upregulated in certain cancer cells under hypoxic conditions. Different from normal gastric tissue, miRNA-373 is upregulated in gastric adenocarcinoma tissue and gastric cancer cell lines. Researchers believe that miRNA-373 acts as an oncogene or tumor suppressor. Studies have also shown that miRNA-373 is associated with osteoarthritis (OA), i.e., the expression of miRNA-373 in OA patients is downregulated, by negatively affecting the regulation of chondrocyte proliferation [12, 13]. miR-373 may be an important target in OA treatment, and the downregulation of miR-373 may become a biomarker for OA detection [14].

The tumor suppressor effect of miRNA-373 has been proven through ovarian cancer research [15]. Zhang et al. [16] found that miRNA-373 can inhibit cell proliferation, migration, and invasion in human bladder cancer cells. Other studies have found that miRNA-373 may be a potential target for treating lung adenocarcinoma and the hepatitis C virus [17–19]. Moreover, miRNA-373 plays a vital role in the pathogenesis of human hepatocellular carcinoma (HCC) and may be a new biomarker for HCC [20–22]. Under hypoxia, miRNA-373 is an HIF-1*α*-dependent miRNA, and it is induced by HIF-1*α*. However, the research on miRNA-373 is still not comprehensive. The time effect of miRNA-specific expression after ischemia is considered to be a useful biological indicator for the clinical diagnosis of brain injury and prognosis. The clinical application of changes in miRNA in human serum has been widely used for the early diagnosis of tumors and other related diseases. Clinically, the disease's severity can be classified according to miRNA expression in children with HIE and subsequently guide clinical treatment [23]. Therefore, miRNA-373 can be used as a new biomarker for the clinical diagnosis of cerebral hypoxia–ischemia and prognosis.

In recent years, the role of HIF-1*α* in the central nervous system has been continuously recognized. Many studies have shown that HIF-1*α* has a protective effect on cerebral hypoxic–ischemic injury. Current studies have also found that HIF-1*α* is involved in pathophysiological processes, such as cerebrovascular disease, nervous system damage, tumors, myocardial ischemia, pulmonary hypertension, preeclampsia, and uterine fetal growth retardation. Baek et al. [24] found that hypoxia can block cell apoptosis. VEGF is one of the most important target genes of HIF-1*α* during hypoxia. VEGF may play an antiapoptotic effect by promoting angiogenesis. Zaman and other experiments proved that HIF-1*α* has an antiapoptotic effect. Yu et al. [25] found that locally injecting adenovirus-mediated HIF-1*α* after brain trauma in rats can promote Bcl-2 expression and inhibit Bax expression, thereby reducing neuronal apoptosis. Other studies on the hypoxic–ischemic model of neonatal rats have shown that EPO can play a neuroprotective effect by inhibiting NMDA receptor-mediated neurotoxicity [26, 27].

Li et al. [28] found that apart from the increased expression of HIF-1*α* in the nucleus, the mRNA and protein levels of EPO and VEGF are also increased in prehypoxic brain tissues, suggesting that HIF-1*α* may withstand cerebral ischemia. MMP-9 is a metalloproteinase that is mainly secreted in zymogen by macrophages, connective tissue cells, and some tumor cells. MMP-9 activity is significantly related to cerebral vascular permeability, blood–brain barrier permeability, and cerebral edema. The level of MMP-9 in the serum of children with HIE is significantly higher than that of the normal control group, indicating that MMP-9 can destroy the basement membrane of blood–brain barrier capillaries, aggravate the capillary permeability of brain tissues, and cause secondary brain edema and brain damage. Serum MMP-9 is an inflammatory marker related to the degree of brain damage and an important indicator for predicting the HIE's prognosis; it has a certain significance for judging the HIE's severity and prognosis. This study's conclusion is consistent with those in the relevant literature.

Here, we found that the HIF-1*α*, VEGF, and MMP-9 protein levels gradually increased from the mild HIE group to the severe HIE group, indicating that hypoxia–ischemia is associated with HIF-1*α*, VEGF, and MMP-9 proteins. Hypoxia–ischemia causes a series of changes in the related factors. The changes in these factors' content can reflect the HIE's severity and provide references for clinical diagnosis and treatment. This study confirmed the increase in HIF-1*α*, VEGF, and MMP-9 levels in the HIE serum samples, which is consistent with those in local and foreign studies.

This study determined that the expression of miRNA-373 gradually increased from the control group to the severe group (*P* < 0.05), suggesting that miRNA-373 can be utilized as a biomarker in the diagnosis and prognosis assessment of HIE. The expression levels of HIF-1*α* also gradually increased from the control group to the mild group to the moderate group. Similarly, the expression level of MMP-9 increased gradually from the control group to the severe group (*P* < 0.01), and it gradually increased from the control group to the mild group to the moderate group to the severe group (*P* < 0.01). The expression level of VEGF increased from the control group to the severe group. These correlations between serum miRNA-373 and HIF-1*α*, between miRNA-373 and MMP-9, and between miRNA-373 and VEGF are all positive, with correlation coefficients of 0.94, 0.92, and 0.945, respectively.

The closer is the correlation coefficient to 1, the stronger is the positive correlation. The correlations' analytical results of the patient (human) sera, i.e., between miRNA-373 and HIF-1*α*, between miRNA-373 and MMP-9, and between miRNA-373 and VEGF, show that the abovementioned four molecules have strong positive correlations. Moreover, when the expression of miRNA-373 increases, the expressions of HIF-1*α*, MMP-9, and VEGF also increase. The expression level of miRNA-373 in the HIE serum samples was higher than that in the control group. The values of HIF-1*α*, MMP-9, and VEGF in the case group were significantly higher than those in the control group. The change in miRNA-373 expression has certain diagnostic significance on neonatal HIE.

In summary, our study explored the changes in the expression of miRNA-373 with respect to HIF-1*α*, MMP-9, and VEGF levels in HIE serum. Our research was able to confirm the value of the miRNA-373 expression in the diagnosis, treatment, and prognosis of HIE. However, the role of miRNA-373 in the pathogenesis of HIE should be further studied. In the occurrence and development of HIE, miRNA-373 is positively correlated with HIF-1*α*, MMP-9, and VEGF. Therefore, the expression of miRNA-373 increases in the occurrence and development of HIE, and HIF-1*α*, MMP-9, and VEGF are all positively correlated. Considering the increase in expression, the present correlation study is conducive as a future research on the mechanism of HIE. miRNA-373 has an extremely complex regulatory effect on the nervous system. Thus, miRNA-373 and specific mechanisms of HIE need to be determined in the future.

## Figures and Tables

**Figure 1:** cDNA agarose gel electrophoresis image. M: marker; 1 and 2: control group; 3–7: severe group; 8–12: moderate group; 13–17: mild group.

**Figure 2:** (a) Amplification curve. (b) Melting curve of miR-373.

**Figure 3:** Fluorescence quantitative PCR to detect the expression of miR-373 in the sample. ^∗^The difference is statistically significant compared with the control group (*P* < 0.05).

**Figure 4:** Comparison of serum HIF-1*α* levels in each group (nmol/mL). ^∗∗^The difference is statistically significant compared with the control group (*P* < 0.01).

**Figure 5:** Comparison of MMP-9 levels in serum of each group (nmol/mL). ^∗∗^The difference is statistically significant compared with the control group (*P* < 0.01).

**Figure 6:** Comparison of serum VEGF levels in each group (nmol/mL). ^∗∗^The difference is statistically significant compared with the control group (*P* < 0.01).

**Figure 7:** Correlation analysis of patient (human) serum miRNA-373 and HIF-1*α*, MMP-9, and VEGF. L: mild group; M: moderate group; S: severe group.

## Data Availability

All data generated or analyzed during this study are included in this article.
